The article "Lactate dehydrogenase D serves as a novel biomarker for prognosis and immune infiltration in lung adenocarcinoma" was retracted in 2024. Reasons: duplicated images; overlap with earlier publications; unreliable results or conclusions.

# Lactate dehydrogenase D serves as a novel biomarker for prognosis and immune infiltration in lung adenocarcinoma

**DOI:** 10.1186/s12885-023-11221-6

**Published:** 2023-08-16

**Authors:** Yu Zhang, Tianyi Zhang, Yingdong Zhao, Hongdi Wu, Qiang Zhen, Suwei Zhu, Shaoshuai Hou

**Affiliations:** 1 Department of Pulmonary and Critical Care Medicine, Shandong Provincial Hospital, Shandong University, Jinan, Shandong 250021 China; 2 Research Center of Translational Medicine, Jinan Central Hospital Affiliated to Shandong First Medical University, Jinan, Shandong 250021 China; 3 Liaocheng Third People’s Hospital, Liaocheng, Shandong 252000 China; 4 Department of Fundamental, Air Force Communications NCO Academy, Dalian, Liaoning 116000 China; 5 College of Pharmacy, Shandong First Medical University, Jinan, Shandong 250021 China; 6 Department of Critical-Care Medicine, Shandong Provincial Hospital Affiliated to Shandong First Medical University, Jinan, Shandong 250021 China; 7 Department of Pharmacy, Tengzhou Central People’s Hospital, Tengzhou, Shandong 277500 China

**Keywords:** Lactate dehydrogenase D, Lung adenocarcinoma, The Cancer Genome Atlas, Biomarker, Prognosis, Immune infiltration

## Abstract

**Background:**

Lung cancer is reported to be the leading cause of death in males and females, globally. Increasing evidence highlights the paramount importance of Lactate dehydrogenase D (LDHD) in different types of cancers, though it’s role in lung adenocarcinoma (LUAD) is still inadequately explored. In this study, we aimed to investigate and determine the relationship between LDHD and LUAD.

**Methods:**

The collection of the samples was guided by The Cancer Genome Atlas (TCGA) datasets and Gene Expression Omnibus (GEO). To ascertain various aspects around LDHD function, we analyzed different expression genes (DEGs), functional enrichment, and protein–protein interaction (PPI) networks. The predictive values for LDHD were collectively determined using the Kaplan–Meier method, Cox regression analysis, and a nomogram. Evaluation of the immune infiltration analysis was completed using Estimate and ssGSEA. The prediction of the immunotherapy response was based on TIDE and IPS. The LDHD expression levels in LUAD were validated through Western blot, qPCR, and immunohistochemistry methods. Wound healing and transwell assays were also performed to illustrate the aggressive features in LUAD cell lines.

**Results:**

The results showed that LDHD was generally downregulated in LUAD patients, with the low LDHD group presenting a decline in OS, DSS, and PFI. Enriched pathways, which include pyruvate metabolism, central carbon metabolism, and oxidative phosphorylation were observed through KEGG analysis. It was also noted that the expression of LDHD expression was inversely related to immune cell infiltration and typical checkpoints. The high LDHD group’s response to immunotherapy was remarkable, particularly in CTAL4 + /PD1- therapy. In vitro studies revealed that the overexpression of LDHD caused tumor migration and invasion to be suppressed.

**Conclusion:**

In conclusion, our study revealed that LDHD might be an effective predictor of prognosis and immune filtration, possibly leading to better choices for immunotherapy.

**Supplementary Information:**

The online version contains supplementary material available at 10.1186/s12885-023-11221-6.

## Introduction

Lung cancer is associated with high incidence and mortality, with lung adenocarcinoma (LUAD) accounting for approximately 40% of all global cases. According to the estimation by the American Cancer Society, about 127,070 people might succumb to lung cancer by the end of 2023, and this translates to 20% of the total cancer mortality [1, 2]. Currently, much has been done with regard to treatment methods for LUAD, considering that development of personalized treatment is underway. Some of the notable developments are the generalization of immune checkpoint inhibitors (ICIs) therapy and target therapy [3]. However, only 20% of locally advanced and metastatic non-small cell lung cancer patients can benefit from immunotherapy. This is explained by the heterogeneity and complexity that is associated with tumors [2]. As a result, the prognosis of LUAD remains poor, leading to a survival rate of around 18% over a period of five years [4]. Therefore, there is an urgent need to identify novel biomarkers that have relatively higher sensitivity and specificity, so that the prognosis of LUAD can be improved.

Tumor cells use glycolysis to satisfy biosynthesis and ATP synthesis, even when adequate oxygen is available and this phenomenon is called the Warburg effect [5, 6]. During this distinctive energy production process by cancerous cells, lactate is formed at a faster rate [6, 7]. Previous reports have emphasized the importance of increasing lactate production, which worsen the prognosis in numerous carcinomas, including lung cancer. Lactate dehydrogenase (LDH) is encoded by LDHA, LDHB, LDHC and LDHD and it is the key tetrameric enzyme that catalyzes the reversible conversion of pyruvate to lactate either aerobically or anaerobically. Accumulating evidence has shed light on the carcinogenic function of LDHA and LDHB in various tumors [8–12]. For example, some studies have highlighted the notion that elevating LDHA levels in papillary thyroid carcinoma can promote tumorigenesis and metastasis via the AMPK signal pathway [13]. It is important to note that only a few studies have focused on the mechanism of LDHD in cancer so far.

Lactate dehydrogenase D (LDHD) is a flavoenzyme that is reportedly located in the mitochondrial [14]. Progressively increasing evidence showed that the expression and function of LDHD is tissue specific. LDHD levels are elevated in prostate cancer and uterine sarcoma, where the flavoenzyme serves as an oncogene [15, 16]. One study reported that the suppression of LDHD in cell renal carcinoma, significantly reduced the overall survival rate of the patients [17]. Currently, the expression and nonenzymatic mechanism of LDHD in LUAD have not been elucidated so it requires further exploration.

This study was conducted to investigate the expression and function of LDHD in LUAD. The results from the analyses of The Cancer Genome Atlas (TCGA) and Gene Expression Omnibus (GEO) showed a reduction in the expression of LDHD in LUAD. Moreover, the Gene ontology (GO), Kyoto Encyclopedia of Genes and Genomes (KEGG) pathway enrichment, and protein–protein interaction (PPI) network analyses were used to evaluate the key genes and signal pathways that are involved in LDHD. The prognostic values of LDHD were assessed done using ROC curves and a nomogram model, based on clinicopathological information. Our study revealed an inverse relationship between immune cell infiltration and LDHD. It is impressive that better response to immunotherapy was observed in the high LDHD group. In vitro, LDHD also contributed to migration and invasion. And the workflow was shown in Fig. 1. This study presents a novel potential biomarker named LDHD, thereby contributing to immune checkpoint inhibitors therapy and the prognosis of tumor. This might contribute to improving the treatment of LUAD.

**Fig. 1:** Flowchart of construction and analysis of LDHD

## Methods

### Data collection

The expression profile of LDHD in pan-cancer was obtained using the TIMER2.0 database (http://timer.cistrome.org/). The transcriptomic data of 516 LUAD and 59 normal samples were collected from The Cancer Genome Atlas (TCGA) (https://portal.gdc.cancer.gov/) database [18]. The RNA-seq data was converted from the FPKM format to the TPM (transcripts per million reads) version for subsequent analyses. Additional normal expression data were obtained from the Genotype Tissue Expression Project (GTEx) (https://www.gtexportal.org) database (*n* = 288). The expression of LDHD was validated using Microarray data from GSE32863, GSE63459, and GSE74706.

### DEGs Between LDHD high expression and low expression Groups in LUAD

The median expression levels of LDHD were used to divide lung adenocarcinoma patients in the TCGA database into two groups as follows: LDHD high-expression group and LDHD low-expression group. The R package DESeq2(1.38.1) [19] was used to determine the expression differences between the two groups. The thresholds for the DEGs were |log_2_-fold change (FC)|> 2.0 and adjusted *p* < 0.05. And the top-10 DEGs was evaluated using a heatmap.

### Functional enrichment analysis

Gene ontology (GO) analysis is a bioinformatics tool for annotating genes and gene-related products. This tool involves three constituents, which are the cellular component (CC), molecular function (MF), and biological process (BP) [20]. The Kyoto Encyclopedia of Genes and Genomes (KEGG) is a collection of databases that are reservoirs for information on genomes, biological pathways, diseases, and chemicals [21]. The Gene set enrichment analysis (GSEA) evaluates the distribution trend of genes that are ranked by phenotype correlation in a gene table, so as to ascertain their role in disease [22]. The R package clusterProfiler (3.14.3) was employed in these functional enrichment analyses [23]. The c2.cp.v7.2.symbols.gmt data set in the Molecular Signature Database (MsigDB) was used as the functional gene set. Each analysis procedure was repeated 1,000 times. Gene sets with *p* < 0.05 and a false discovery rate (FDR) < 0.05 were considered to be significantly enriched gene sets.

### Protein–protein Interaction network

The protein–protein interaction (PPI) network of DEGs with threshold value | log_2_FC |> 2.0 was constructed using Search Tool for the Retrieval of Interacting Genes (STRING, https://string-db.org/) online database. The top-10 HUB genes were evaluated using the MCC algorithm of CytoHubba in Cytoscape (version 3.7.2) [24]. The top 50 binding proteins that interacted with LDHD were obtained from the STRING database, and the set parameters were as follows: minimum required interaction score ("medium confidence (0.400)") and active interaction score ("experiment, text mining, database"). The Cytoscape software (version 3.7.2) was used to visualize protein interactions, while the top-10 Hub genes were assessed using the CytoHubba plug-in.

### Survival analysis

Kaplan–Meier survival analyses of all clinicopathological characteristics were undertaken in LUAD patients, with the *p* values being calculated by the log-rank test. The curve cut-point function of the survminer package (0.4.9) in R was employed in classifying the patient expression data into either low or high LDHD expression. Univariate and multivariate Cox regression were then used to identify independent prognostic factors [25]. *p* < 0.05 represented statistical significance.

### Construction and validation of a prognostic nomogram

An overall survival prediction nomogram that was time-dependent was developed based on the analyses of the Cox proportional hazards regression, which consisted of independent risk factors. ROC curves were created and calibration was done to assess the fitness of the nomogram. The area-under-the-curve (AUC) usually ranged between 0.5 and 1. As shown in the calibration figure, there was a 45-degree line that served as an ideal line. The closer the time-dependent and ideal lines were the better the predictive ability of the nomogram [26]. The nomogram and calibration plot were generated by the RMS package (version 6.2–0) and survival package (version 3.2–10) was for predicting OS [27]. Time-dependent ROC analysis at 1-, 3-, and 5-year was performed using the R package time ROC (0.4).

### Immune infiltration analysis and estimation of sensitivity to immunotherapy

The immunescore was calculated by the estimation algorithm using the "Estimate" R package (1.0.13) [28]. The single sample gene set enrichment analysis (ssGSEA) algorithm served as a tool for evaluating the relative enrichment of infiltrating immune cells in LUAD. Samples from the gene expression profile of each tumor quantify the relative concentration of each type of immune cell grading, completed by the GSVA R package (1.34.0) [29]. The Spearman correlation analysis was used to investigate the correlation between LDHD expression and immune cells. Variations in immune infiltration levels between the LDHD high and low expression groups were determined using the Wilcoxon rank sum test. Further analysis was done on the correlation between LDHD and the immune checkpoints PD1, PD-L1, CTLA4, LAG3, TIM3, and TIGIT [30]. The immunotherapeutic effect and immune escape based on the expression of LDHD were predicted from the Cancer Immunome Atlas (TCIA) (http://tcia.at/) and Tumor immune Dysfunction and Exclusion (TIDE) database (http://tide.dfci.harvard.edu/) [31, 32].

### Lung adenocarcinoma samples and immunohistochemistry (IHC)

Six pairs of primary lung cancer tissues and noncancerous tissues were collected from patients who underwent surgery. It was confirmed that these patients were never subjected to radiotherapy or chemotherapy prior to surgery. Clinical and pathological evidence confirmed lung cancer in all the patients who participated in the study. All the procedures in this study were approved by the Ethics Committee of Liaocheng Third People’s Hospital (NO.2023002), and informed consent was obtained from all participants before surgery. Tissue slides were prepared and deparaffinized by baking them in an oven at 65℃ for 2 h. They were then dewaxed using gradient ethanol. Goat serum was used for blocking and slides were then stained with an LDHD antibody (1:250, ProteinTech, 14,398–1-AP) overnight, at 4℃. The samples were then incubated together with secondary antibodies (Goat anti-rabbit antibody, Zhongshan Biotechnology Co, Beijing, China) for an hour, at room temperature. DAB staining, hematoxylin redyeing, and hydrochloric acid alcohol differentiation were then done on the samples, respectively. The images were captured using an Olympus microscope imaging system (Olympus, Tokyo, Japan).

### Cell culture and treatment

The human lung epithelial cells (BEAS-2B) were obtained from the American Type Culture Collection (ATCC, Manassas, VA) and were cultured in DMEM medium (Gibco, United States) that was supplemented with 10% fetal bovineserum (Gibco, United States), penicillin (100 U/ml), and streptomycin (100 mg/ml, Gibco, United States), in a humidified atmosphere with 5% CO_2_, at 37^◦^C. Human lung cancer cell lines (H1299, A549, H838, H1975) were purchased from Procell Life Science and Technology Co. Ltd. (Wuhan, China) and were cultured in RPMI-1640 (Gibco, United States), which was supplemented with 10% fetal bovine serum (Gibco, United States) at 37 °C, in a humidified atmosphere with 5% CO_2_.

### siRNAs and plasmids

Both LDHD siRNAs and plasmid were conducted by RiboBio (Guangzhou, CN). siRNA sequences are as follows: LDHD siRNA1 5’-GGAAGAGUGCAGCCGGCUACA-3’, LDHD siRNA2 5’- ACUGCAUCCUGCUGGUCAACC -3’, LDHD siRNA3 5’- AGGAGAUAGUCCAGCAGAACG-3’. Cells were seeded in six-well plates for approximately 24 h before transfection. Ribo FECT™ CP Transfection KIT (C10511-05, RiboBio) and Lipofectamine 3000 (L3000-015, Invitrogen) were used according to the instructions.

### Western blotting

Cells were incubated together with the RIPA lysis buffer (Solarbio Biotechnology, Beijing, China) and the quantified protein lysates were separated on 12% PAGE mini-gels. A one-hour electroblotting procedure was then carried out to transfer the protein into 0.45 µm PVDF membranes (Millipore, United States). Membranes were blocked in TBST which contained 5% non-fat milk for an hour before incubating in primary antibodies at 4^◦^C, overnight. Rabbit anti-LDHD antibody (1:1000, ProteinTech, 14,398–1-AP) and rabbit Beta Actin antibody (1:2500, Protein Tech, 20,536–1-AP) were used as primary antibodies. The membranes were then incubated with the corresponding second antibody (goat anti-rabbit IgG) prior to detection with enhanced chemiluminescence reagents (ECL, Millipore, United States).

### Real-time polymerase chain reaction

RNA was extracted using the TRIzol Reagent (Invitrogen, United States) according to the manufacturer’s instructions. First strand cDNA synthesis was performed using the Revert Aid First Strand cDNA Synthesis Kit (Thermo scientific). The real-time polymerase chain reaction (RT-qPCR) was carried out using the Ultra SYBR Mixture kit (Cwbio, CW2601M) on Roche 480II as follows: first, 95^◦^C for 2 min until denaturation took place; second, 40 cycles at 95^◦^C for 15 s, 60^◦^C for a minute; third, 95^◦^C to allow for melting; and last, 50^◦^C for 30 s to allow for cooling down. The synthesized strands were as follows: 5'-AGGAGATAGTCCAGCAGAAC-3' (forward) and 5'-TTCAGATCCTCCTTGGTCTG-3' (reverse) for LDHD and 5'-GAAGTGTGACGTGGACATCC-3' (forward) and 5'-CCGATCCACACGGAGTACTT-3 (reverse) for β-actin.

### Immunofluorescence staining

Cells were seeded on chamber slides before they were treated for 48 h. Mitochondrial staining was done by incubating the cells with 100 nM MitoTracker Red CMXRos (Molecular Probes) at 37 °C, for 30 min. Then, the cells were fixed with 4% paraformaldehyde, washed with PBS three times for five minutes, permeabilized in 0.1% Triton X-100, and then blocked for an hour with 1% goat serum (Solarbio, SL038). Incubation with an LDHD primary antibody (1:250, ProteinTech, 14,398–1-AP) overnight at 4 °C was then done. This was followed an hour’s incubation with the secondary antibody Alexa Fluor®-488 (1:1000, Invitrogen), at 37 °C. A counterstaining procedure for the nuclei was done using Hoechst 33,342 (Life technologies, H3570). The slides were mounted with the fluorescent mounting medium (Dako). The fluorescent images were taken with the Nikon microscope imaging system (Olympus, Tokyo, Japan) and Image J was used to analyze them.

### Wound-healing assay

Cells were seeded in six-well plates at a density of 4 × 10^5^ cells per well. Once the cells reached 95% confluence, a cell monolayer was scrapped with a sterile 200 μl pipette tip to create a wound area. The detached cells were washed off with PBS. Cells that migrated to the wounded region were observed by a M7000 (100 × magnification) immediately and after 12 h. The experiments were performed in triplicates.

### Transwell assays

Transwell assays were performed using the BD chambers (8-mm pores; BD Biosciences, Shanghai, China). About 1 × 10^5^ cells per well were seeded in the upper chamber, followed by culturing in a serum-free medium. A medium with 30% serum was placed in the lower chambers. The cells migrated through the Transwell membrane, and they were fixed with 4% paraformaldehyde prior to being stained with crystal violet (Solarbio, Beijing, China). The difference between the migration and invasion assays was that the Transwell chambers for the former was not coated with Matrigel while those for the latter were. All Transwell treatments were conducted in triplicates.

### Statistical analysis

All statistical analyses were carried out using R (3.6.3). Statistical significance was analyzed using the Wilcoxon rank-sum and paired sample t-test. The correlation between clinical characteristics and LDHD expression was evaluated using the Wilcoxon rank-sum test and univariate logistic regression. Univariate and multivariate Cox regression analysis were used for prognostic analysis. Spearman correlation and Wilcoxon rank-sum test were used to analyze the immune signature of LDHD in LUAD. In all analyses, *p* < 0.05 was considered statistically significant. *p < 0.05, **p < 0.01, and ***p < 0.001.

## Results

### LDHD expression was downregulated in LUAD

A sum of 33 cancer types were screened by TIMER2.0 to investigate the mRNA expression of LDHD (Fig. 2A). Substantial discrepancies in gene expression in 16 of the 33 cancer types were observed, from which a decreasing LDHD trend was noted in most tumor tissues, except for kidney renal clear cell carcinoma (KIRC). This study focused on the differences in LDHD levels in lung adenocarcinoma. After combing relevant data from GTEx and TCGA, we found LDHD expression was decreased in tumor tissues, which was also observed in 58 paired tissues (Fig. 2B, C). Furthermore, the lower expression of LDHD was validated in GSE32863, GSE63459, and GSE74706 (Fig. 2D-F). The clinicopathological differences between the high and low expression groups of LDHD were also found, including primary therapy outcome and number pack years smoked (Table 1). Overall, the obtained results suggested the potential application of that LDHD as a diagnostic biomarker in LUAD.

**Fig. 2:** Expression levels of LDHD in different types of tumors and lung adenocarcinoma. **A** Differential expression of LDHD in pan-cancer samples from the TIMER2.0 database; **B** LDHD expression in lung adenocarcinoma and non-matched normal tissues in the TCGA and GTEx databases; **C** LDHD expression in lung adenocarcinoma and matched normal tissues in the TCGA databases; **D**-**F** The LDHD mRNA expression between LUAD and normal tissues based on data from GSE32863 (**D**), GSE63459 (**E**), and GSE74706 (**F**) dataset. TCGA, The Cancer Genome Atlas; GTEx, Genotype Tissue Expression Project; *p < 0.05, **p < 0.01, and ***p < 0.001

**Table 1:** Correlation of LDHD and clinicopathological parameters in patients with lung adenocarcinoma

Characteristics	Low expression of LDHD	High expression of LDHD	*P* value
n	258	258	
Pathologic T stage, n (%)			0.085
T1	74 (14.4%)	95 (18.5%)	
T2	151 (29.4%)	127 (24.8%)	
T3&T4	31 (6%)	35 (6.8%)	
Pathologic N stage, n (%)			0.253
N0	158 (31.3%)	174 (34.5%)	
N1	52 (10.3%)	44 (8.7%)	
N2&N3	43 (8.5%)	33 (6.5%)	
Pathologic M stage, n (%)			0.649
M0	169 (45.4%)	178 (47.8%)	
M1	11 (3%)	14 (3.8%)	
Pathologic stage, n (%)			0.344
Stage I	130 (25.6%)	146 (28.7%)	
Stage II	64 (12.6%)	58 (11.4%)	
Stage III & Stage IV	60 (11.8%)	50 (9.8%)	
Primary therapy outcome, n (%)			**0.029**
PD&SD	62 (14.5%)	43 (10%)	
CR&PR	151 (35.3%)	172 (40.2%)	
Gender, n (%)			0.724
Female	137 (26.6%)	141 (27.3%)	
Male	121 (23.4%)	117 (22.7%)	
Race, n (%)			0.336
White	201 (44.8%)	188 (41.9%)	
Asian& Black or African American	27 (6%)	33 (7.3%)	
Age, n (%)			0.968
< = 65	120 (24.1%)	119 (23.9%)	
> 65	130 (26.2%)	128 (25.8%)	
Residual tumor, n (%)			0.545
R0	168 (46.4%)	177 (48.9%)	
R1&R2	7 (1.9%)	10 (2.8%)	
Anatomic neoplasm subdivision, n (%)			0.757
Left	99 (19.8%)	102 (20.4%)	
Right	152 (30.3%)	148 (29.5%)	
Number pack years smoked, n (%)			**0.029**
< 40	80 (22.8%)	94 (26.8%)	
> = 40	102 (29.1%)	75 (21.4%)	

### Functional enrichment of DEGs and LDHD-related genes

The differential expression genes (DEGs) in LDHD-high and LDHD-low patients were presented by heatmap and volcano map, with 39 being upregulated and 72 being downregulated (Fig. 3A-B). The relationships between total DEGs and top-10 genes is shown in Supplementary Fig. 1 and Supplementary Table 1. The results from the functional enrichment analyses revealed that DEGs were enriched in the maintenance of nucleosome morphology and DNA replication process, both of which affect cell proliferation (Fig. 3C, Supplementary Table 2). In particular, the G2/M checkpoint and histone acetyltransferase (HATs) pathways were also enriched, which were bound up with tumorigenesis and immune response (Fig. 4A-F, and Supplementary Table 3). Besides, interacting proteins that are associated with LDHD were screened out using the STRING database. After CytoHubba plugin analyses in Cytoscape, top-10 hub genes were selected, and the majority of these genes were reported to be related with various cancers (Fig. 5A-B). The findings from GO and KEGG analyses further confirmed the vital effects of LDHD in cancer, as pyruvate metabolism and aerobic respiration were collected (Fig. 5C-D and Supplementary Table 4).

**Fig. 3:** Results of differentially expressed gene (DEG) and functional enrichment analysis.** A** Volcano plot of DEGs (red: upregulation; blue: downregulation); **B** Heatmap of the correlation between LDHD expression and the top 10 DEGs; **C** GO and KEGG analysis of DEGs; DEGs, differentially expressed genes, GO, Gene ontology, BP, Biological process, CC, Cellular component, MF, Molecular function. KEGG, Kyoto Encyclopedia of Genes and Genomes; ^*^p < 0.05, ^**^p < 0.01, and ^***^p < 0.001

**Fig. 4:** Results of GSEA enrichment analysis of DEGs(**A**-**F**); GSEA, Gene set enrichment analysis

**Fig. 5:** Protein–protein interaction (PPI) network, GO analysis and KEGG analysis of 50 LDHD targeted binding proteins.** A** Protein–protein interaction network; **B** Top 10 hub genes of PPI network; **C**-**D** Visualization network for GO and KEGG analysis of PPI network; PPI, Protein–protein interaction

### The prognostic value of LDHD in LUAD

To assess the prognostic values of LDHD, the survival curves were generated using Kaplan–Meier methods. The lower-expression LDHD group presented a significantly worse OS, DSS and PFI than the high-expression group (Fig. 6A-C). Analysis of 11 patient subgroups according to clinicopathological features were also conducted, such as age, gender, subdivision, smoking information, race, process after primary theory and pathologic grade. The obtained results indicated that patients with low LDHD had significantly worse OS, DSS, and PFI in most clinical subgroups (Supplementary Figure S2-3). These results suggest that LDHD is an effective and protective prognostic factor for LUAD.

**Fig. 6:** Prognostic value of different expression of LDHD in lung adenocarcinoma evaluated by Kaplan–Meier survival analysis. **A** OS, Overall Survival; **B** DSS, Disease Specific Survival; **C** PFI, Progress Free Interval

### Establishment and validation of a prognostic nomogram

To enhance prediction of the prognosis in LUAD patients, a nomogram that combined LDHD and clinical information was developed. After univariable and multivariable Cox regression analysis, three factors were incorporated into the nomogram, and these are the primary theory outcome, residual tumors, and LDHD expression level (Fig. 7A-C and Table 2). The prediction accuracy of the nomogram was compared by time-dependent ROC and calibration curves. AUCs for one-, three- and five-year OS prediction of the risk factors were 0.732, 0.752, and 0.690, respectively (Fig. 7D). The calibration also validated a good performance of the prediction of the nomogram (Fig. 7E). The results suggested that the nomogram was a suitable prognostic model for LUAD patients.

**Fig. 7:** Establishment and visualization of clinical prognostic prediction model of LDHD in LUAD.** A**-**B** Forest plot of OS in LUAD based on the univariate and multivariate Cox regression. **C** Construction of a prognostic nomogram figure. **D** Time-dependent ROC analysis. **E** Calibration curves for the nomogram of 1-, 3- and 5-year survival probability. ROC, Receiver operating characteristic

**Table 2:** Univariate analysis of LDHD and clinical parameters with overall survival rate

Characteristics	Total(N)	Univariate analysis		Multivariate analysis	
		**HR (95% CI)**	***P* value**	**HR (95% CI)**	***P* value**
T stage (T2&T3&T4 vs. T1)	504	1.665 (1.182—2.345)	0.002	1.369 (0.838—2.238)	0.210
N stage (N1&N2&N3 vs. N0)	495	2.582 (1.922—3.470)	< 0.001	1.574 (0.824—3.006)	0.170
M stage (M1 vs. M0)	363	2.143 (1.251—3.672)	0.006	1.334 (0.670—2.657)	0.412
Pathologic stage (Stage II&III&IV vs. Stage I)	499	2.958 (2.177—4.021)	< 0.001	1.475 (0.738—2.948)	0.271
Primary therapy outcome (PR&CR vs. PD&SD)	421	0.354 (0.252—0.499)	< 0.001	0.289 (0.174—0.482)	** < 0.001**
Residual tumor (R1&R2 vs. R0)	353	3.991 (2.227—7.152)	< 0.001	2.876 (1.391—5.948)	**0.004**
Gender (Male vs. Female)	507	1.070 (0.800—1.431)	0.648		
Age (> 65 vs. < = 65)	497	1.213 (0.904—1.629)	0.198		
Race (White vs. Asian& Black or African American)	449	1.447 (0.884—2.368)	0.123		
Anatomic neoplasm subdivision (Right vs. Left)	493	1.032 (0.764—1.394)	0.838		
Number pack years smoked (> = 40 vs. < 40)	345	1.038 (0.723—1.490)	0.840		
LDHD (High vs. Low)	507	0.712 (0.531—0.954)	0.023	0.728 (0.495—0.968)	**0.031**

### Immunoinfiltration analysis of lung adenocarcinoma

Immune cells take an important part in tumor microenvironment, which are closely related to tumor development, immunotherapy and prognosis in tumor patients. In this study, we used Estimate and ssGSEA to determine the differences in immune infiltration. The results showed negative correlation between LDHD expression and the immuneScore (Fig. 8A). Significant differences in expression were shown by ssGSEA in 14 immune cells. It is important to note that immunosuppressive cells (Tregs and Th2) were highly expressed in the low LDHD group (Fig. 8B-C). The results from the Spearman correlation analysis were displayed in Fig. 8C and Supplementary Figure S4.

**Fig. 8:** Correlation between LDHD expression and immune infiltration in lung adenocarcinoma. **A** Relationship between immune score and LDHD expression in patients with lung adenocarcinoma; **B** Correlation between LDHD expression and relative abundance of 24 kinds of immune cells in patients with lung adenocarcinoma. The size of the point corresponds to the absolute value of Spearman's rank correlation coefficient; **C** Comparison of immune infiltration levels of 24 immune cell types in patients with lung adenocarcinoma in groups with high and low LDHD; DCs, dendritic cells; aDCs, activated DCs; iDCs, immature DCs; pDCs, plasmacytoid DCs; Th, T helper cells; Th1, type 1 Th cells; Th2, type 2 Th cells; Th17, type 17 Th cells; Treg, regulatory T cells; Tgd, T gamma delta; Tcm, T central memory; Tem, T effector memory; Tfh, T follicular helper; NK, natural killer; ^*^p < 0.05, ^**^p < 0.01, and ^***^p < 0.001

### Expression of immune checkpoint genes and assessment of sensitivity to immunotherapy

Classic emerging immune checkpoint genes were analyzed in the low and high LDHD groups. Interestingly, the included genes were highly expressed in the low LDHD group (Fig. 9A). Based on the relationship between LDHD and immune checkpoint genes, the sensitivity of LUAD patients to the immune checkpoint blockade (ICB) therapy was further explored. TIDE is a web platform that works by modeling tumor immune dysfunction and exclusion, in order to predict ICB clinical response. The high LDHD group seemingly showed better sensitivity to immunotherapy, as shown by the higher immunotherapy responder rate, TIDE score, and exclusion score (Fig. 9B-D). The immunophenoscore (IPS) further validated the fact that high LDHD tumor was associated with high immunogenicity and that the high LDHD group might benefit from the CTAL4 + /PD1- therapy (Fig. 9E-H).

**Fig. 9:** Signature of immune co-inhibitors and immune response in LUAD based on LDHD expression. **A** Heatmap of correlation between LDHD expression and the immune checkpoints; **B**-**D** TIDE signatures predict the immune response of LUAD patients in LDHD low and high groups; **E**–**H** The comparison of Immunophenoscore (IPS) containing CTLA4-/PD1-, CTLA4-/PD1 + , CTLA4 + /PD1- and CTLA4 + /PD1 + were constructed in different groups of LDHD expression; *p < 0.05, **p < 0.01, and ***p < 0.001

### LDHD was lowly expressed and influenced the migration and invasion in LUAD

First, LDHD expression was detected in six pairs of LUAD tumor tissues and adjacent normal tissues by IHC. Compared to the corresponding non-cancerous tissues, the cancer ones exhibited lower LDHD expression (Fig. 10A). Furthermore, Western blotting and qPCR confirmed that LDHD protein and mRNA levels in various human LUAD cell lines were lower in normal lung cell (Fig. 10B). As a member of the lactate dehydrogenase family, LDHD is distributed in the mitochondria of A549 cells (Fig. 10C). After the differential expression of LDHD, the effect on migration and invasion were detected in LUAD cells. Upregulation of LDHD could inhibit the migration and invasion in A549 and H1975 cells (Fig. 10D-G). While in the LDHD silencing group, the ability of H1299 and H838 to invade and migrate were significantly higher (Fig. 11).

**Fig. 10:** LDHD is differentially expressed and LDHD overexpression restrains the migration and invasion of H1975 and A549 cells. **A** Representative images from immunohistochemistry staining of LDHD in lung cancers (*n* = 6). Scale bars are in the pictures. **B** Levels of LDHD in the indicated lung cancer cell lines and normal cell were measured by a western blot assay. LDHD mRNA expressions in listed lung cancer cells and normal cell were shown, and results were quantified. **C** Immunofluorescent staining was used to detect location of LDHD in A549 cells. **D** RT-qPCR and western blot showed the over-expression of LDHD in A549 and H1975. **E**–**F** Transwell assays showed that LDHD overexpression inhibited lung cancer cells mobility and metastasis. **G** Wound healing assay was performed to show the effect of LDHD overexpression on migration of H1975 and A549 cells. A strach wound was made on cell surface and cells were photographed at 0 h, 12 h. Representative pictures are shown. *p < 0.05, **p < 0.01, and ***p < 0.001

**Fig. 11:** LDHD knockdown promotes the migration and invasion of H1299 and H838 cells. **A** RT-qPCR and western blot analysis were used to detect the knockdown efficiency of LDHD in H1299 and H838 cells. **B**-**C** Transwell assays showed that LDHD knockdown could enhance the invasion and metastasis of H1299 and H838 cells. **D** Wound healing assay was performed to show the effect of LDHD knockdown on migration of H1299 and H838 cells. Representative images are shown. *p < 0.05, **p < 0.01, and ***p < 0.001

## Discussion

Lung cancer is a deadly disease globally, with LUAD accounting for nearly 40% [3]. In recent years, increasing awareness of the immune escape mechanism led to the revolutionization of the treatment landscape of lung cancer through ICIs [33]. However only 20–40% of all patients will respond to ICI therapy and even fewer will have long-term disease remission [34]. This study proposed a simple but robust biomarker called LDHD, which was downregulated in LUAD patients, consistent with a suppression-expression in kidney tumors [17]. To the best of our knowledge, the current study is the first to identify the prominent decrease, biological function, and immune landscape of LDHD in LUAD patients.

Functional analyses showed that DEGs and LDHD-related genes were mainly enriched in the G2/M cell cycle and pyruvate metabolism. Zhang *et.al* showed that the inhibition of LDHA suppresses tumor growth by promoting the arrest of the G2/M cell cycle and apoptosis via the JNK signal [35]. Tumor cells prefer gaining ATP from aerobic glycolysis (an important feature of metabolic reprogramming), during which pyruvate is reduced to lactate in an LDH-driven reaction [36]. Increasing aerobic glycolysis provided more energy for the tumor cells, thereby immensely contributing to tumorigenesis, metastasis, and drug resistance [37]. Therefore, the assumption that LDHD might participate in tumor growth, migration, and invasion was brought forward in this study. Interestingly, the experiments carried out latter validated our notion by showing that the elevation of LDHD could suppress migration and invasion of A549 and H1975 cells.

Lactate was regarded as a bridge between metabolic reprogramming and immune escape, yet it was previously considered a waste byproduct during aerobic glycolysis [38]. Increasing evidence show that lactate can acidify the tumor microenvironment (TME) and then exert immunosuppressive actions and promote tumor invasion, which is associated with immune escape [39]. Tumor-infiltrating immune cells are typical cells in TME. It is worth noting that different subsets of immune cells play various roles that contribute to anti-tumor effects. They can even skew into opposite phenotypes in response to stimulation by lactate [40]. Tumor-associated macrophages can sense the presence of lactate, and then stimulate M2 polarization, thereby causing immunosuppression and proliferation of tumor cells [41]. Tregs play an important role in immune suppression and maintenance of an immune balance. Lactate can serve as fuel for Tregs so as to promote growth and suppressive function [42]. As an isoform of LDH, LDHD catalyzes the reversible conversion of pyruvate to lactate, in addition to helping in the elimination of methylglyoxal, a cytotoxic byproduct in glycolysis [16]. In line with these findings, prediction was made that LDHD might exert a synergistic effect on tumor escape through lactate.

This study further clarified the relationship between LDHD and prognosis, where suppressed LDHD expression was associated with worse prognosis. Furthermore, LDHD expression was represented as an independent protective factor by the univariable and multivariable Cox regression analysis. Truth be told, a single factor can’t provide a comprehensive and accurate assessment of the tumor prognosis, which is why a nomogram that contained LDHD expression and some important clinical information was employed. The ROC and calibration curves showed good efficacy of the prognostic model that was built [43]. Therefore, there was convincing evidence that LDHD was a negative independent predictor of prognosis.

As we mentioned earlier, immune cells with tumor microenvironment play diverse roles in immune surveillance. Here, ssGSEA revealed that the LDHD low-expression group had higher enrichment of Th2 cells and Tregs, which exhibit tumor-promoting activities. Cytokines like IL-4 and IL-13, produced by Th2 cells, can polarize macrophages into M2 cells, which hamper anti-tumor immune response [44]. In tumor cells, the anti-tumor efficacy of effector T-cells can be retarded by Tregs as the upregulation of co-inhibitory receptors, including cytotoxic T-lymphocyte-associated antigen-4 (CTLA-4), programmed cell death protein 1 (PD-1), T-cell immunoglobulin and mucin-domain containing-3 (TIM-3) and lymphocyte activation gene-3 (LAG-3). These receptors can cause T-cells to become exhausted [40]. Previous reports found that NSCLC patients who have higher levels of Treg or Th2 cells had a worse prognosis, and this possibly explains the poor prognosis in the LDHD low-expression group [45, 46]. Clinical guidelines introduced immune checkpoint inhibitors (ICIs) treatment as the first-line therapy for patients with metastatic non-small cell lung cancer (NSCLC), without oncogenic driver alterations [2]. The TIDE score and IPS were evaluated to investigate whether LDHD can partly guide the medicine plan for ICIs therapy [47]. Based on the results from this study, a conclusion was made that the LDHD high group might benefit from ICIs therapy more, especially in CTLA4 + treatment, although the opposite group had higher expression of immune checkpoints. Apart from PD-1 or CTLA4 signaling, other inhibitory signals also promote immune tolerance [30]. So, when one immune checkpoint was blockaded, other negative factors were still existed, playing anti-tumor effect. This may explain the poor efficacy of a single ICI treatment in LDHD low group.

LDHD was mainly located in inner membrane of mitochondria [16]. We also detected its location in A549 cells through immunofluorescence assays, and this was consistent with the previous report. In view of the above-mentioned potential functions, it was proposed that LDHD might influence tumor progress by regulating mitochondrial metabolism, which then promotes migration and invasion.

Although our study improved the current understanding of LDHD in LUAD, there are still some limitations to take note of. First, the data that was obtained from TCGA and GEO were limited and mainly focused from Western countries, so it may poorly represent Asian countries. Second, the validation of the nomogram was not conducted by an external database. Finally, specific investigation of the underlying mechanism of LDHD was not undertaken. Therefore, further study should be taken to explore the particular action mechanism of LDHD in LUAD.

## Conclusion

Our study is the first to investigate the expression and potential function of LDHD in LUAD. Bioinformatics analysis revealed that the low-expression group of LDHD had a worse prognosis and was negatively linked to immune infiltration and immune checkpoint expression. LDHD might function as a suppression gene by regulating energy metabolism and TME, thereby constraining immune evasion. Patients with high expression of LDHD might be more sensitive to ICI therapy. In vitro, the elevation of LDHD can impair migration and invasion of LUAD cells. In summary, this work provided evidence in support of the predictive and immune effect of LDHD in LUAD patients.

### Supplementary Information

**Additional file 1: Supplementary Figure 1.** Protein–protein interaction (PPI) network of LDHD-related DEGs and top 10 hub genes. **Supplementary Figure 2.** Prognostic value of different expression of LDHD in lung adenocarcinoma evaluated by Kaplan–Meier survival analysis in different subgroups. **Supplementary Figure 3.** Prognostic value of different expression of LDHD in lung adenocarcinoma evaluated by Kaplan–Meier survival analysis in different subgroups. (A-G) DSS survival curves of age≤65, Male, smoker, Anatomic neoplasm subdivision (Right), N0, M0, Stage I and Stage II; (H-Q) PFI survival curves of age (＞65 and ≤65), gender (Male and Female), smoker (Yes and No), Anatomic neoplasm subdivision (Right), N0, M0, Stage I and Stage II; DSS, Disease Specific Survival; PFI, Progress Free Interval. **Supplementary Figure 4.** Correlation between LDHD expression and immune infiltration levels in LUAD(A-W).

**Additional file 2: Supplementary Table 1.** Top 10 upregulated and 10 downregulated LDHD-related DEGs. **Supplementary Table 2.** Gene Ontology (GO) and KEGG pathway functional enrichment of LDHD-related DEGs. **Supplementary Table 3.** Gene set enrichment analysis (GSEA) enrichment analysis of DEGs. **Supplementary Table 4.** GO analysis and KEGG analysis of 50 LDHD targeted binding proteins.

**Additional file 3.**

## Data Availability

The data used during this current study are available in TCGA database (https://portal.gdc.cancer.gov/), GTEx database (http://www.gtexportal.org/home) and GEO database (https://www.ncbi.nlm.nih.gov/geo/).

## Abbreviations

LDHD: Lactate dehydrogenase D
LDH: Lactate dehydrogenase
LUAD: Lung adenocarcinoma
NSCLC: Non-small cell lung cancer
TCGA: The Cancer Genome Atlas
GTEx: Genotype Tissue Expression Project
DEGs: Differentially expressed genes
GO: Gene ontology
KEGG: Kyoto Encyclopedia of Genes and Genomes
GSEA: Gene set enrichment analysis
PPI: Protein-protein interaction
OS: Overall Survival
DSS: Disease Specific Survival
PFI: Progress Free Interval
ROC: Receiver operating characteristic
CR: Complete response
PR: Partial response
SD: Stable disease
PD: Progressive disease
HR: Hazard ratios
CI: Confidence intervals
OR: Odds Ratio
KICH: Kidney Chromophobe
DCs: Dendritic cells
aDCs: Activated DCs
iDCs: Immature DCs
pDCs: Plasmacytoid DCs
Th: T helper cells
Th1: Type 1 Th cells
Th2: Type 2 Th cells
Th17: Type 17 Th cells
Treg: Regulatory T cells
Tgd: T gamma delta
Tcm: T central memory
Tem: T effector memory
Tfh: T follicular helper
NK: Natural killer
RT-qPCR: Real-time quantitative polymerase chain reaction
IHC: Immunohistochemistry
